The article "Effect of Application of Treadmill Training on Metabolic Control and Vitamin D Level in Saudi Patients with Type 2 Diabetes Mellitus" was retracted in 2023. Reason: concerns about the peer review.

# Effect of Application of Treadmill Training on Metabolic Control and Vitamin D Level in Saudi Patients with Type 2 Diabetes Mellitus

**DOI:** 10.1155/2022/3059629

**Published:** 2022-01-30

**Authors:** Ahmad El Askary, Alaa Shafie, Mazen Almehmadi, Hatem H. Allam, Lamiaa K. Elsayyad, Asmaa F. Hassan, Bader B. Althobaiti, Mohamed Mansour Khalifa, Tamer Saber, Aisha H. Alharthi, Amal F. Gharib

**Affiliations:** ^1^Department of Clinical Laboratory Sciences, College of Applied Medical Sciences, Taif University, P.O. Box 11099, Taif 21944, Saudi Arabia; ^2^Department of Physical Therapy, College of Applied Medical Sciences, Taif University, P.O. Box 11099, Taif 21944, Saudi Arabia; ^3^Department of Medical Physiology, College of Medicine, Taif University, P.O. Box 11099, Taif 21944, Saudi Arabia; ^4^Department of Clinical Laboratories, King Abdulaziz Specialist Hospital in Taif, Ministry of Health, Taif, Saudi Arabia; ^5^Department of Human Physiology, Faculty of Medicine, Cairo University, Egypt; ^6^Department of Human Physiology, College of Medicine, King Saud University, Saudi Arabia; ^7^Department of Internal Medicine, Faculty of Medicine, Zagazig University, Zagazig, Egypt

## Abstract

**Background:**

Diabetes mellitus type 2 and vitamin D deficiency are both prevalent in the Saudi Arabia. Vitamin D deficiency treatment with supplements carries a risk of intoxication.

**Aim:**

The present study is aimed at elucidating the effect of exercise on modulation of metabolic status and vitamin D level in patients with type 2 diabetes mellitus (T2DM).

**Methods:**

A sum of 110 type 2 diabetic patients were voluntarily enrolled for the present investigation by dividing them into two separate groups (55 individuals for each group), the diabetic study group and diabetic control group. The diabetic study group was engaged in the training program using treadmill exercise. Laboratory parameters were monitored before and after the training program.

**Results:**

There were significant elevation in the diabetic study group compared to diabetic control group regarding postexercise vitamin D level, high-density lipoprotein (HDL) (*p* value ≤ 0.001, 0.045; respectively). In addition, triglycerides, low-density lipoprotein (LDL), glycosylated hemoglobin (HbA1C), and homeostatic model assessment-insulin resistance (HOMA-IR) were significantly decreased (*p* value < 0.001 for all mentioned parameters). Moreover, there were significant higher level in postexercise parameters as compared to preexercise level in the diabetic study group.

**Conclusion:**

The exercise training program improved the metabolic control and vitamin D level after three months of intervention.

The article "Effect of Application of Treadmill Training on Metabolic Control and Vitamin D Level in Saudi Patients with Type 2 Diabetes Mellitus" was retracted in 2023. Reason: concerns about the peer review.

## 1. Introduction

Recently, deficiency of vitamin D represents a significant risk to human health in industrialized world [1]. In Saudi Arabia, hypovitaminosis D was detected in 60% of Saudi populations. Being sunny country, the deficiency of vitamin D is still prevalent in different ages and more common in females [2]. The estimation of 25-hydroxyvitamin D [25(OH) D] from serum is considered as major significant marker for evaluation of vitamin D status in human body [3]. Low vitamin D level is believed to be caused by inactivity, chronic illnesses, diabetes mellitus, and obesity. Other factors, which may influence low vitamin D level in human body, may be caused by genetics [4, 5]. The prevalence of type 2 diabetes mellitus (T2DM) has increased notably over the world [6]. The global prevalence of T2DM has been estimated to reach approximately 422 million which may reach about 552 million adult human beings by year 2030 [7]. The prevalence of diabetes mellitus (DM) in Saudi Arabia is rapidly elevated and became the most prevalent health problem in last 20 century owing to remarkable change in the population lifestyle [8].

Vitamin D receptors (VDR) have been detected in a variety of human cells, including pancreatic and insulin-responsive cells called adipocytes. Adipose tissues in human body are major storehouse of vitamin D and a main supplier of inflammatory adipokines and cytokines [9]. Several recent research have been conducted to connect mediators of inflammatory response with level of vitamin D in people suffering from T2DM. Vitamin D has a direct influence on endothelial function and is an essential anti-inflammatory and antioxidant agent [10–12]. Moreover, vitamin D is integral for calcium and phosphorus homeostasis, as along with blood glucose control. Vitamin D will help T2DM patients in reducing their risk of fractures and can improve muscle atrophy and blood sugar level [13, 14].

Obesity, particularly visceral obesity, is considered as one of the most well-known risk factors for prevalence of T2DM. The concomitance of vitamin D deficiency and obesity has also been established as a possible link between prevalence of diabetes and obesity [15]. Vitamin D deficiency was related to a lower quality of life and compliance with diabetes treatment [16]. Vitamin D supplementation or medicinal vitamin D therapy holds potential benefit in prevention or treatment of diseases as DM is still debatable. According to epidemiological and association reports, vitamin D deficiency is related to higher risk of both types of DM [17].

Researchers have examined the impact of regular exercise on cardiovascular and metabolic illnesses, including diabetes. Exercise has become an important therapy option for glucose metabolic disorders because it stimulates glucose transporter 4 (GLUT4) in skeletal muscle as an adaptive response independent of insulin [18, 19].

The article "Effect of Application of Treadmill Training on Metabolic Control and Vitamin D Level in Saudi Patients with Type 2 Diabetes Mellitus" was retracted in 2023. Reason: concerns about the peer review.

High-intensity exercise has been shown to increase insulin sensitivity and glucose tolerance (above 85% of maximal aerobic capacity) [20, 21]. The activity of vitamin D and VDR expression has been shown to be affected by mechanical stress during exercise, such as HIIT [18, 22].

Little is known about the effect of exercise on vitamin D levels in T2DM. As a result, the present research sought to determine the impact of frequent exercise on serum vitamin D levels.

## 2. Materials and Methods

### 2.1. Study Population

A case-control study was conducted involving voluntare 110 Saudi patients with T2DM. This study was performed in College of Applied Medical Sciences at both Departments of Physical Therapy and Clinical Laboratories in Taif University, Saudi Arabia. Diagnosis of T2DM was established as per criteria established by American Diabetes Association in 2013 [23]. The age, sex, and body mass index (BMI) [24] were noted down for all participants.

Included participants were followed up for 3 months starting from January 2021 till the end of March 2021. The patients were divided into two equal groups (55 subjects for each), involving diabetic study and diabetic control groups. The exclusion criteria were patients with type 1 diabetes, metabolic syndrome, mal-absorptive states, gestational diabetes, any musculo-skeletal disorders, acute or chronic infections, cancer, pregnancy, and lactation. In addition, all subjects included in present investigation did not intake vitamin D or calcium supplementation in the last three months. All subjects were collected from distinct private and public hospitals in Taif city, Western Area, Saudi Arabia. Prior to enrollment, consent was taken from participants through clarification of study aim.

## 3. Methods

### 3.1. Sampling and Biochemical Analysis

Blood samples were collected from all participants of both groups, i.e., diabetic study and diabetic control groups before entering the study and from type 2 diabetic study group after 12 weeks of aerobic exercise. Fasting venous blood (5 mL) was collected under complete aseptic conditions and divided into two tubes: plain tubes for serum separation to assay 25(OH)D, blood glucose, lipid profile, and EDTA treated tubes for glycosylated hemoglobin (HbA1c) and insulin measurements and stored at -20°C till utilization for further analysis. The level of 25(OH)D in blood samples from all subjects was determined using an Abcam human vitamin D ELISA kit (USA) (Cat no: ab213966) following manufacturer instructions. Individuals with vitamin D serum level of <20 ng/ml were perceived as deficient.

The article "Effect of Application of Treadmill Training on Metabolic Control and Vitamin D Level in Saudi Patients with Type 2 Diabetes Mellitus" was retracted in 2023. Reason: concerns about the peer review.

Fasting blood glucose (FBG), total cholesterol (TC), triglycerides (TG), and high density lipoprotein-cholesterol (HDL-C) levels were analyzed using enzymatic colorimetric techniques according to Trinder [25], Allain et al. [26], Lopes-Virella et al. [27], and Glick et al. [28], respectively, utilizing kits purchased from ELI Tech Group (Puteaux, France). LDL-C was estimated as suggested by Friedewald et al. [29]. HbA1c was analyzed using automated glycosylated hemoglobin analyzer (Bio-Rad, USA).

The plasma samples were utilized to determine fasting insulin concentration measured with an electrochemiluminescence immunoassay (Elecsys, Roche, Switzerland).

Homeostasis model for insulin resistance (insulin HOMA-IR) was determine using following equation, [Insulin (uUml − 1) + blood glucose (mmoll − 1)] = HOMA − IR 22.5 [30].

### 3.2. Physical Therapy Methods

#### 3.2.1. Calculation of Exercise Intensity

The heart rate zone was calculated using the Martti Karvonen algorithm. Initially, each participant heart rate at rest (rest-HR) was determined by requesting to wear heart rate monitor and lay down in a prone posture in noise-free room for 10 minutes. The maximal heart rate (max-HR) was then estimated using the formula: max − HR = 220 − age. The heart rate reserve (HRR) was estimated using following formula: HRR = max − HR–rest − HR. Lastly, target heart rate (target-HR) was determined as follows: target − HR = HRR × intensity percent + rest − HR. The moderate-intensity exercise with a heart rate of 50% to 70% was applied [31].

#### 3.2.2. The Intervention

The study group's participants were present at the physical therapy lab, and intervention was in the form of treadmill aerobic exercises (T-AE) that were applied for three times per week till three months for the study group [32]. A motorized treadmill was used to induce exercises, whereas each session was started with 5 minutes of warming up further consists of stretching of lower limb muscles and was ended after 5 minutes cooling down. Training program for the study group followed the sequence illustrated in (Table 1). The inclination was 5° up. The treadmill speed was set at 2.5 mills/hour at start, then raised by 0.5 mill/h each with 1 minute unless the target rate was achieved.

The hand rails were permitted to be grasped by the participants in order to preserve balance adjustment. The exercise sessions were monitored by the principal investigator and one helper in order to achieve high precision and protection measures.

### 3.3. Statistical Analysis

Statistical analysis was done using SPSS version 20 (SPSS Inc., Chicago, Illinois, USA). Within-subject and between-subject serum level variations were determined using the repeated measure MANOVA test and Bonferroni pairwise comparisons before and after the intervention was undertaken, respectively. The results were considered statistically significant at *p* value < 0.05 and highly significant at *p* value < 0.001.

The article "Effect of Application of Treadmill Training on Metabolic Control and Vitamin D Level in Saudi Patients with Type 2 Diabetes Mellitus" was retracted in 2023. Reason: concerns about the peer review.

## 4. Results

The criteria of subjects included in the present study are represented in (Table 2). There were no statistically significant difference in age, BMI, gender, and level of physical activity between diabetic study and control groups. In the diabetic study group, there were 26 females (47.3%) and 29 males (52.7%), whereas in the diabetic control group, there were 28 females (50.9%) and 27 males (49.1%). The difference between the two groups was statistically nonsignificant (*p* value = 0.703).

In addition, the preintervention laboratory results displayed, the diabetic study and diabetic control groups had no significant differences as shown in (Table 3).

Regarding the postintervention laboratory data of studied groups, results indicated significant increase in for vitamin D level, HDL (*p* value ≤ 0.001, 0.045; respectively) in diabetic study group as compared to the control group during postexercise. On the other hand, triglycerides, LDL, glycosylated hemoglobin, and HOMA-IR were significantly decreased (*p* value < 0.001 for all mentioned parameters) (Table 4).

The laboratory data in the diabetic study group indicated a significant mean in postintervention when compared to preintervention (Table 5).

## 5. Discussion

T2DM is a chronic disease characterized by insulin resistance and cell dysfunction, which eventually lead toward change in insulin secretion [33]. The vitamin D supplementation and circuit exercise were supposed to aid during treatment of diabetes in aged people with deficient vitamin D level. Trials to validate the effectiveness of the difficult operation are still lacking [34]. Within the study diabetic group, there was highly significant mean in posttreatment as compared to pretreatment. (post-vitamin D; posttotal cholesterol; posttriglycerides; post- LDL; postfasting glucose; post-HbA1c%; postfasting insulin; post-HOMA-IR). Previously, it was reported that vitamin D intake can improve insulin release and sensitivity [35]. In general, vitamin D intake has shown lower LDL-C and TG levels [36], while increase in HDL-C [37]. Moreover, exercise-induced increases in vitamin D-VDR axis may improve lipid profiles through different mechanisms as suggested by Chaudhuri et al. [38].

Blood glucose levels in T2DM patients may be influenced by a number of factors; exercise (mode, time, length, frequency, and intensity), diet, and clinical characteristics, i.e., age, sex, baseline metabolic control, and duration of diabetes [39]. Exercise training that improves physical activity has shown substantially reduction for abdominal fat tissue. Bacchi et al. [40] found that after 16 weeks of aerobic exercise on a treadmill or bike, the visceral and subcutaneous fat areas of the abdomen were greatly decreased. Regular physical exercise has been shown to regulate blood glucose, enhance physical ability of patients, and reduce the development of T2DM [41]. Muscle mass increased with most forms of exercise on a physiological level, resulting in an increase in basal metabolic rate and overall capacity for glucose and fat oxidation. Finally, the structure of muscle fiber types is adjusted depending on the activity type [42]. In the presence of insulin, physical exercise improves insulin sensitivity in the liver, resulting in decreased glucose synthesis and output. As a result, exercise is widely regarded as one of the most effective nonpharmacological treatments for nonalcoholic fatty liver disease, hypertriglyceridemia, and hepatic insulin resistance [41, 43].

The article "Effect of Application of Treadmill Training on Metabolic Control and Vitamin D Level in Saudi Patients with Type 2 Diabetes Mellitus" was retracted in 2023. Reason: concerns about the peer review.

The American Diabetes Association (ADA) recommended moderate-intensity aerobic exercise for 150 minutes or high-intensity aerobic exercise for 75 minutes in each week for patients with T2DM [41]. Way et al. [44] reported regardless of exercise intensity, and the influence of exercise on insulin sensitivity remained for 2 to 3 days. Another study discovered that exercising at a moderate-high level for at least 12 weeks may increase mitochondrial activity rather than exercising at a lower intensity [45]. Sung and Bae [46] reported total cholesterol and triglycerides were significantly lowered in diabetic elderly men who walked for 50 minutes three times a week with 65-75% of their maximum heart rate for 24 weeks. In a separate study, Umpierre et al. [47] reported after meta-analysis, aerobic exercise, independent of kind, intensity, time, or quantity of training are helpful in decreasing insulin resistance. Therefore, by promoting fatty acid oxidation and reducing insulin levels, aerobic exercise decreases the insulin resistance index.

Physical exercise and improvement of blood vitamin D levels have been correlated in previous studies, which might be owing to extended vitamin D metabolism or higher sunlight exposure [18]. Wanner et al. [48] found that those who exercised outside had substantially elevated levels of 25(OH) D compared to individuals exercised indoors. Saremi et al. [49] reported that vitamin D supplement, and doing aerobic activities simultaneously had a positive impact on lowering cardiovascular risk factors, rising insulin sensitivity, and lowering insulin resistance. In addition, aerobic exercise improves blood glucose levels and lipid profile. Moreover, both insulin and exercise can enhance glucose absorption from the intracellular to the cell surface through glucose transporter (GLUT4) in exercised muscles [50]. The 25(OH) D level in patients with type II diabetes may increase if took vitamin D supplemented with aerobic exercises or only the vitamin D as supplement [51]. It is noteworthy to mention, in type 2 diabetic patients, elevated levels of 25(OH) D were recorded as compared to the control group.

The article "Effect of Application of Treadmill Training on Metabolic Control and Vitamin D Level in Saudi Patients with Type 2 Diabetes Mellitus" was retracted in 2023. Reason: concerns about the peer review.

The current study demonstrated the impact of exercise training on the metabolic regulation and vitamin D status of patients with type 2 diabetes, and it may serve as a guide for developing better programs that prevent the negative effects of utilizing medications. This research has some limitations: the number of included subjects was small, and we did not use different exercise intensities in this study.

## 6. Conclusion

The current study revealed that the exercise training program improved the metabolic control and vitamin D level after three months of intervention. Therefore, the outcomes of the present investigation can be forwarded to relevant authorities to consider for individuals experiencing low vitamin D conditions.

## Figures and Tables

**Table 1:** The progression of moderate-intensity treadmill aerobic exercises (T-AE).

Week	Intensity %	Time (min)
1, 2	50%	20
3, 4	55%	25
5, 6	60%	30
7, 8	65%	35
9, 10	70%	40
11, 12	70%	40

**(a):** 

Multivariate test					
	Value	*F*	Hypothesis df	Error df	Sig
Wilks' lambda	0.968	1.781	2.000	107.000	0.173

**(b):** 

Bonferroni pairwise comparisons				
Demographic variables	Diabetic study group Mean ± SD	Diabetic control group Mean ± SD	Mean diff. diabetic study–diabetic control	Significance
Age (year)	47.95 ± 5.08	46.47 ± 5.05	1.48	0.130
Sex				
Female	26	28	1.23	0.703
Male	29	27		
BMI percentile	28.31 ± 3.35	27.65 ± 3.47	0.66	0.316

**Table 3:** Bonferroni pairwise comparisons for preintervention laboratory data between-subjects included in the study.

Laboratory data	Diabetic study group (*n* = 55)	Diabetic control group (*n* = 55)	*p* value
Previtamin D ng/ml	19.53 ± 5.81	20.12 ± 6.51	0.617
Pretotal cholesterol (mg/dl)	263.62 ± 50.05	259.98 ± 44.21	0.687
Pretriglycerides (mg/dl)	352.45 ± 73.95	348.20 ± 46.20	0.718
Pre-LDL-C (mg/dl)	185.27 ± 42.01	179.35 ± 30.23	0.398
Pre-HDL-C (mg/dl)	32.27 ± 7.58	34.98 ± 10.49	0.123
Prefasting glucose (mg/dl)	272.76 ± 64.83	267.93 ± 52.62	0.668
Pre-HbA1c (%)	11.25 ± 2.46	10.84 ± 1.28	0.268
Prefasting insulin (*μ*IU/mL)	20.02 ± 2.06	20.13 ± 2.15	0.786
Pre-HOMA-IR	9.38 ± 2.16	9.85 ± 2.12	0.250

The article "Effect of Application of Treadmill Training on Metabolic Control and Vitamin D Level in Saudi Patients with Type 2 Diabetes Mellitus" was retracted in 2023. Reason: concerns about the peer review.

**Table 4:** Bonferroni pairwise comparisons for postintervention laboratory data (between-subjects).

Laboratory data	Diabetic study group (*n* = 55)	Diabetic control group (*n* = 55)	*p* value
Postvitamin D (ng/ml)	24.97 ± 6.66	20.17 ± 6.64	<0.001^∗∗^
Posttriglycerides (mg/dl)	162.05 ± 47.38	348.40 ± 45.73	<0.001^∗∗^
Post-LDL-C (mg/dl)	144.67 ± 30.79	179.38 ± 29.66	<0.001^∗∗^
Post-HDL-C (mg/dl)	39.16 ± 10.86	35.02 ± 10.55	0.045^∗^
Postfasting glucose (mg/dl)	169.49 ± 55.34	268.13 ± 52.57	<0.001^∗∗^
Post-HbA1c (%)	7.54 ± 1.37	10.85 ± 1.35	<0.001^∗∗^
Postfasting insulin (*μ*IU/mL)	15.85 ± 2.03	20.15 ± 2.29	<0.001^∗∗^
Post-HOMA-IR	5.49 ± 1.43	9.91 ± 2.20	<0.001^∗∗^

^∗^ *p* value < 0.05 S; ^∗∗^*p* value < 0.001 HS.

**Table 5:** Bonferroni pairwise comparisons for Laboratory data (within-subjects) in patients group.

Laboratory data	Diabetic study group (*n* = 55)		Bonferroni	
	Preintervention	Postintervention	Mean diff.	*p* value
Vitamin D ng/ml	19.53 ± 5.81	24.97 ± 6.66	-5.436	<0.001^∗∗^
Total cholesterol (mg/dl)	263.62 ± 50.05	227.87 ± 48.40	35.745	0.002^∗^
Triglycerides (mg/dl)	352.45 ± 73.95	162.05 ± 47.38	190.400	<0.001^∗∗^
LDL (mg/dl)	185.27 ± 42.01	144.67 ± 30.79	40.600	<0.001^∗∗^
HDL (mg/dl)	32.27 ± 7.58	39.16 ± 10.86	-6.891	0.002^∗^
Fasting glucose (mg/dl)	272.76 ± 64.83	169.49 ± 55.34	103.273	<0.001^∗∗^
HbA1c (%)	11.25 ± 2.46	7.54 ± 1.37	3.713	<0.001^∗∗^
Fasting insulin (*μ*IU/mL)	20.02 ± 2.06	15.85 ± 2.03	4.164	<0.001 ^∗∗^
HOMA-IR	9.38 ± 2.16	5.49 ± 1.43	3.891	<0.001 ∗∗

^∗^ *p* value < 0.05 S; ^∗∗^*p* value < 0.001 HS.

## Data Availability

Data are available from the corresponding author upon request.
